# LncRNA GAS5 Suppresses Colorectal Cancer Progress by Target miR-21/LIFR Axis

**DOI:** 10.1155/2022/3298939

**Published:** 2022-08-24

**Authors:** Juan Xie, Jing-Jing Wang, Ya-Jun Li, Jia Wu, Xiao-Jing Gu, Xiao-Rong Yang

**Affiliations:** Department of Gastroenterology, General Hospital of Ningxia Medical University, Ningxia 750004, Yinchuan, China

## Abstract

GAS5 is abnormally high in colorectal cancer tissues, which is a specific expression of lncRNA in colorectal cancer (CRC). Nevertheless, its biological function in CRC has not been elucidated. The abnormal high expression of GAS5 in CRC is the specific expression of lncRNA in CRC. The purpose of our study is to explore the effect of GAS5 on CRC and its mechanism. The expression of GAS5 in 53 paired normal and colorectal cancer tissues and colorectal cancer cell lines was detected by real-time PCR. The biological effects of GAS5, miR-21, and LIFR were measured by functional assays, including wound healing, transwell assays, and in vivo assays. We ensured the carcinogenesis role of GAS5 in CRC in the xenograft nude model. The dual-luciferase reporter assay system and chromatin immunoprecipitation method were used for target evaluation and Western blot for verification. GAS5 was significantly decreased in tumor tissues and CRC cells, and the low expression of CAS5 in CRC promoted tumor metastasis and decreased the survival of patients. GAS5 knockdown increases the cell viability, inhibits apoptosis, and promotes migration. Xenografted tumors in nude mice studies showed that GAS5 knockdown promoted tumor growth and caused worse lesions in colorectal. Furthermore, GAS5 increases the expression level of target gene LIFR to promote the apoptosis of CRC cells by binding to miR-21. Our study revealed that a novel pathway about lncRNA GAS5 inhibited the proliferation and metastasis of CRC cells by targeting miR-21/LIFR which provides a new strategy to treat CRC.

## 1. Introduction

Long noncoding RNA (lncRNA) is a transcription product with a length of more than 200 nucleotides with limited coding potential. LncRNAs can be located in nuclear or cytosolic fractions [1]. Harrow J et al. reported that human lncRNAs contain 13870 lncRNA genes that produce 23898 lncRNAs [2]. The abnormality of lncRNAs plays an important role in the occurrence and development of human diseases. LncRNAs may play the role of oncogenes or tumor suppressor genes in tumor, regulating many important characteristics of tumors, such as proliferation, apoptosis, autophagy, and tumor metastasis [3]. One study showed that lncRNA is secreted to extracellular cells in the form of exosomes [4]. LncRNA in body fluids has the potential of a biomarker, indicating the progress and malignancy of tumors and guiding personalized treatment [5].

Colorectal cancer (CRC) is one of the most common tumors in China. Most of the patients are in advanced stage at the time of consultation because of its occult onset [6]. More than 1 million individuals will develop colorectal cancer each year, and the disease-specific rate is nearly 33% in the world [7]. The formation of colorectal cancer includes genetic and epigenetic changes, in which the abnormal expression of lncRNA plays an important role [8]. At present, hundreds of oncogenes and antioncogenes have been discovered, but the function and mechanism of these genes are still unclear [9]. As a newly discovered research hotspot, lncRNA has important research value. Differentially expressed lncRNA in colon cancer is likely to be an important cancer-promoting or anticancer factor and a new tumor marker in colorectal cancer [10, 11].

GAS5 is a specific expression of lncRNA in colorectal cancer, which is abnormally high in colorectal cancer tissues [12, 13]. Much research has proved that lncRNAs are involved in diverse biological processes [14, 15]. The abnormal expression of lncRNA GAS5 has been found in multiple tumors, and lots of research studies have shown that GAS5 could affect many cellular processes, such as cell proliferation and apoptosis [14–16]. Lu found that compared with normal pancreatic tissues, the expression of GAS5 in pancreatic cancer decreased significantly [14]. Overexpression of GAS5 could inhibit cell proliferation [14]. But the relationship between GAS5 and prostate cancer is still unclear. This study aimed to investigate the effect and mechanism of GAS5 in colorectal cancer. Researchers have found that leukemia inhibitory factor receptor (LIFR) plays an important role in the inhibition of tumorigenesis [15, 16]. In HCC tumor tissues, LIFR was significantly reduced by increased hypermethylation of its promoter [17, 18]. Therefore, these suggest that LIFR as a biomarker of tumor progression is more effective in assessing prognosis [19].

In this study, we studied the biological function of GAS5 in colorectal cancer and explored the potential mechanisms of cell migration, metastasis, and invasion mediated by GAS5. The data indicate that GAS5 directly targets miR-21/LIFR. Our research provides new evidence to support a new regulatory pathway where GAS5 plays a key role in tumor metastasis and invasion.

## 2. Methods and Materials

### 2.1. Patients and Tissue Samples

The research subjects were 53 patients with CRC in China (Table 1). We have got the consent of all the patients. From March 2019 to July 2020, these patients underwent radical resection of primary colorectal cancer in general surgery of the General Hospital of Ningxia Medical University. The criteria for inclusion in the patient cohort included a unique pathological diagnosis of colorectal cancer; surgical resection, defined as the removal of all tumor nodules by histological examination without cancer at the cutting edge; and complete clinicopathological data. This study was reviewed and approved by the Ethics Committee of the General Hospital of Ningxia Medical University (Ningxia, China).

### 2.2. Cell Culture and Reagents

The CRC cell line and a colorectal cell line were obtained from the Shanghai Institute of Cell Biology, Chinese Academy of Sciences (Shanghai, China). The cells grew in Dulbecco's modified Eagles medium (DMEM, GIBCO-BRL, Invitrogen), which was added with 10% heat inactivation fetal bovine serum (FBS) and antibiotics and was incubated at 37°C with 5% CO_2_.

### 2.3. Western Blot

The whole cell lysates were prepared with detergent buffer. According to the manufacturer's manual (Beyotime Institute of Biotechnology, Shanghai, China), protein concentration was determined by the BCA protein assay. The same amount of (50 *μ*g) protein was isolated by 10% sodium dodecyl sulfate-polyacrylamide gel electrophoresis (SDS-PAGE) and transferred to a PVDF membrane (Millipore, Billerica, MA). The PVDF membrane was incubated overnight at 4°C with diluted 1 : 10000 diluted antiglyceraldehyde3-phosphate dehydrogenase (GAPDH, Sigma) and antibodies cleaved caspase-3 (1 : 500), LIFR (1 : 500) (Cell Signaling Technology, Beverly, MA). After incubation with 1 : 1000 diluted anti-immunoglobulin horseradish peroxidase binding antibody for 1 hour, immunocomplexes were detected by enhanced chemiluminescence (Cell Signaling Technology).

### 2.4. RNA Extraction and Reverse Transcription-Quantitative Polymerase Chain Reaction (RT-qPCR)

The relative gene expression of GAS5 and GAPDH and the expression level of miR-21 and U6 snRNA were analyzed according to the previous method [20]. The only difference was the primers, as given in Table 2.

### 2.5. Dual-Luciferase Reporter Assay

The binding sites between GAS5 and miR-21 were predicted by DIANA. A GAS5 fragment containing the predicted wild-type (WT) or mutant (MUT) miR-21 binding site was generated and inserted into luciferase report vector PSI-CHECK-2 (Promega, Shanghai, China). 293T cells were placed on 24-well plates and grew to 80% confluence. The cells were then cotransfected with 100 ng miR-21 mimics or NC, 50 ng GAS5-WT or GAS5-MUT plasmids, and 5 ng pRL-CMV containing Renilla luciferase using Lipofectamine 2000. The luciferase activity was detected by the Dual-Luciferase® reporter assay system, at 48 hours after transfection. Luciferase activity and Renilla luciferase activity were normalized in each group.

### 2.6. Cell Viability Assay

Cell viability assay was measured according to the previous method [20]. The cells were cultured in Dulbecco's modified Eagle's medium with 10% fetal bovine serum at 37°C in a humidified atmosphere containing 5% CO_2_, for cell viability assay.

### 2.7. Apoptosis Analysis

Cell apoptosis was analyzed according to the previous method [21].

### 2.8. Transwell Assays

Cells were transfected with GAS5 and/or miR-21 for 48 h; then, 10000 cells in serum-free medium were reseeded in the upper wells of chambers. The lower chambers contained medium with 10% fetal bovine serum. Transwell assays were detected according to the previous method that Lu et al. used [21].

### 2.9. In Vivo Tumor Study

These female BALB/C nude mice (purchased from Beijing Vital River Laboratory Animal Technology Co., Ltd.) were used in this experiment. These mice (6/group) were housed under barrier conditions in individually ventilated microisolation caging, with autoclaved cage, food, water bottles, and bedding. Direct injection of SW480 cells have different GAS5 expression status into colonic mucosa of 5-week-old female BALB/C nude mice (seven mice each group) under direct vision. When the bodyweight of the mouse decreased significantly and cachexia was found, the mice was killed by breaking their necks, the abdominal cavity was examined, and the tumor formation and metastasis in the abdominal cavity were observed.

### 2.10. Statistical Analyses

The derived values are expressed as the means ± SD. A single factor analysis of variance (ANOVA) was used to compare the mean among multiple groups, and a multiple-range least significant difference (LSD) was used for intergroup comparisons. *P* < 0.05 was considered statistically significant. SPSS 21.0 software was used for statistical analysis.

## 3. Results

### 3.1. Low Expression of CAS5 in Colorectal Cancer (CRC) Promotes the Tumor Metastasis and Decreases the Survival of Patients

To explore the role of GAS5 in the development of CRC, we first investigated the expression of GAS5 in 53 colorectal cancer (CRC) patient's specimens. We found that GAS5 was significantly downregulated in colorectal cancer specimens (Figure 1(a)) and in metastasis specimens (Figure 1(b)) compared with adjacent nontumor/nonmetastasis tissues. Furthermore, patients with lower GAS5 level exhibited shorter overall survival (OS) (*P*=0.0273) and worse disease-free survival than those with higher GAS5 level (Figure 1(c)). Moreover, expression levels of GAS5 were decreased in all examined colorectal cancer cells, as compared to NCM460 normal colon mucosal cells (Figure 1(d)).

### 3.2. Knockdown of CAS5 Increases Cell Viability, Inhibits Cell Apoptosis, and Promotes Cell Migration

To further explore the biological roles of GAS5, a series of functional experiments were carried out. A siRNA targeting GAS5 was used to inhibit the expression of GAS5 (siGAS5). Real-time qPCR was used to detect GAS5 in colorectal cancer cells (Figure 2(a)). Inhibition of GAS5 expression can significantly increase cell viability, and GAS5 upregulation obviously promotes apoptosis in CRC (Figure 2(b)). Flow cytometry analyzed the apoptosis rates of the transfected CRC at cells 72 h. GAS5 upregulation obviously promoted apoptosis in CRC cells (Figure 2(c)). Transwell assays were carried out to assess the invasion capability of CRC cells transfected with GAS5, siGAS5, and NC at 72 h. The capacity of migration in CRC was also significantly inhibited by GAS5 upregulation, and inhibition of GAS5 expression also significantly promoted the migration of colorectal cancer cells (Figure 2(d)). Western blot assays were carried out to determine the expression of cleaved caspase-3 in the transfected CRC cells at 72 h. Inhibition of GAS5 expression also significantly weakens the expression of cleaved caspase-3 in CRC cells (Figure 2(e)).

### 3.3. Knockdown of CAS5 Promotes the Tumor Growth and the Lesion of Colorectal in the Animal Model

Direct injection of SW480 cells has different GAS5 expression status into colonic mucosa of 5-week-old female BALB/C nude mice (seven mice each group) under direct vision. Tumor weights for the nude mice were detected. The detection of weight showed that the weight of xenograft tumors with SW480 cells inhibitory expressing GAS5 was higher than that of the control group (Figure 3(a)). The tumor formation and metastasis in the abdominal cavity were observed. As shown in Figure 3(b), GAS5 overexpression displayed less formation of tumor in the abdominal cavity when compared with untreated mice. On the contrary, siGAS5 enhanced formation of tumor and cause bodyweight loss in animals (Figures 3(b)–3(d).

### 3.4. GAS5 Is Suppressed by miR-21 in Tumor Cells to Promote the CRC

LncRNAs could combine with miRNAs directly and have the function of a molecular sponge. We explored whether GAS5 has similar functions. Bioinformatics analysis showed that miR-21 possesses more binding sites in GAS5 than other miRNAs, and miR-21 was upregulated in CRC tissues, which inhibited tumor progression in CRC cells. Therefore, miR-21 is chosen as the further research object. The putative binding sites between GAS5 and miR-21 are shown in Figure 4(a). Compared with NCM460 normal colon mucosal cells, miR-21 expression level was decreased in all examined CRC cells (Figure 4(b)). The results of qRT-PCR showed that miR-21 expression level in CRC cells transfected with siGAS5 increased compared with NC cells (Figure 4(c)). The results of the dual-luciferase reporter assay showed that the cells cotransfected with GAS5-WT and miR-21 mimic showed low luciferase activity, while the cells cotransfected with GAS5-MUT and miR-21 mimics have not significantly inhibited on luciferase activity (Figure 4(d)). To further explore the biological effects of GAS5 and miR-21, a series of functional experiments were carried out. As shown in Figure 4(e), the overexpression of GAS5 significantly inhibited the proliferation of CRC cells, the upregulation of miR-21 significantly weakened the inhibition induced by GAS5 overexpression, and the reduction of microRNA-21 significantly reduced the cell viability (Figure 4(e)). Western blot was used to detect the expression of caspase-3 in the transfected CRC cells at 72 h. High expression of GAS5 and inhibiting the expression of miR-21 significantly enhances the expression of cleaved caspase-3 in CRC cells (Figure 4(f)). Flow cytometry analyzed the apoptosis rates of the transfected CRC cells at 72 h. High expression of GAS5 and inhibiting the expression of miR-21 obviously promoted apoptosis in CRC cells (Figure 4(g)). Transwell assays were carried out to assess the invasion capability of CRC cells transfected at 72 h. The capacity of migration in CRC was also significantly inhibited by high expression of the GAS5 group and inhibiting the expression of the miR-21 group, whereas miR-21 overexpression evidently inversed the effect of GAS5 upregulation (Figure 4(h)).

### 3.5. GAS5 Binds with miR-21 to Promote LIFR to Suppress the Tumor Cells

miRNA has the ability to directly bind to mRNA and function as inhibiting protein expression. The analysis of the 3′-UTR of LIFR mRNA revealed the potential binding sites for miR-21, which implied the existence of a regulative relationship between miR-21 and LIFR (Figure 5(c)). Dual-luciferase reporter assays were performed to prove miR-21 regulation of LIFR. miR-21 markedly decreased the luciferase activity of wide-type LIFR 3′-UTR in CRC cells, whereas the suppression effect was abrogated after the 3′-UTR binding site of LIFR was mutated (Figure 5(d)). Next, real-time PCR analysis showed an increased LIFR expression level in miR-21 inhibitor cells and a decreased LIFR level in miR-21 overexpressing cells. Correspondingly, LIFR protein levels coincided with the change of mRNA levels in NC and GAS5-miR-21 overexpressing cells (Figures 5(e), 5(f)).

To further explore the cell biological roles of GAS5, miR-21, and LIFR, a series of functional experiments were carried out. As shown in Figure 6(a), LIFR overexpression significantly constrained the viability of CRC cells. On the contrary, the cell viability was significantly higher than NC by inhibiting the expression of LIFR. However, the cell activity in NC was consistent with that in GAS5+siLIFR and miR-21+LIFR (Figure 6(a)). Meanwhile, flow cytometry analyzed the apoptosis rates of the transfected CRC at cells 72 h. Overexpression of LIFR obviously promoted apoptosis in CRC cells. On the contrary, inhibiting the expression of LIFR obviously decreased the percentage of apoptosis cells in CRC cells (Figure 6(b)). Transwell assays were carried out to assess the invasion capability of CRC cells transfected at 72 h. The capacity of migration in CRC was also significantly inhibited by overexpression of the LIFR group and inhibiting the expression of LIFR obviously promoted capacity of migration, whereas GAS5 overexpression evidently inversed the effect of LIFR downregulation (Figure 6(c)). As shown in Figure 6(d), LIFR upregulation also significantly enhanced the expression of cleaved caspase-3 in CRC cells. The expression of cleaved caspase-3 in CRC cells was significantly reduced by inhibiting the expression of LIFR, whereas GAS5 and miR-21 overexpression evidently inversed the effect of siLIFR downregulation (Figure 6(d)).

## 4. Discussion

In the last five years, a great number of research studies were focused on the study of growth arrest-specific transcript 5 (GAS5), a long noncoding RNA, which were found to play an important role as a tumor suppressor in many cancers, such as gastric cancer [21], ovarian cancer [22], cervical cancer[23], and esophageal squamous cell [24]. GAS5 was first found to fail to express in differentiation cells but could be ubiquitously expressed during embryo development and in adult life in a mouse model [25]. Then, GAS5 was found to be aberrantly expressed in many cancers and diseases, and the abnormal expression affected the biological characteristics of them [26, 27], including cell proliferation [28], tumor growth [29], and metastasis [30]. The biological function of GAS5 was complex, and it depends on the type of cancers and the targets in the downstream. In colorectal cancer (CRC), with the third highest morbidity, GAS5 plays a cruel role for the cancer prognosis [28, 31]. The GAS5 was found to be a promising prognostic biomarker of colorectal metastases for early stage CRC patients because of the significantly different expression between colorectal metastases and primary tumors [32].

In our current study, we found that the expression of GAS5 in tumor tissues was significantly lower than in adjacent tissues in CRC, and it was the same for some human colon cancer cell lines when compared with the normal. It was consistent with the results described as Yang in their study [33]. The low expression of CAS5 in CRC promoted the tumor metastasis and decreased the survival of patients. Furthermore, knockdown of GAS5 could increase cell viability, inhibit cell apoptosis, and promote the migration of cells. The results in xenografted tumors in nude mice showed that the knockdown of GAS5 could promote tumor growth and cause worse lesions in colorectal. Based on these findings, we indicated that the low expression of GAS5 in tumor cells promoted the biological progression of CRC.

The miR-21 was detected to high expressing in primary tumor tissues and colorectal metastasis tissues of CRC patients [34, 35]. We predicted that lncRNA GAS5 had a complementary sequence pairing with miR-21, and GAS5 acted as a competing endogenous RNA (ceRNA) to inhibit miR-21 to bind to target mRNA and repress the biological functions of it. Subsequently, we found that the expression level of miR-21 in human colon cancer cell lines was lower than the normal cell lines and knockdown of GAS5 could increase the expression level of miR-21, and GAS5 could bind with miR-21 in vivo. According to the results, we considered that the interaction between GAS5 and miR-21 would affect the function of each other on CRC. Interestingly, the overexpression of GAS5 could significantly suppress the expression of miR-21, and the overexpression of GAS5 and miR-21 caused a higher cell viability than the former. Meanwhile, the inhibition of miR-21 and overexpression of GAS5 promoted the apoptosis and suppressed the migration of cells. All results indicated that GAS5 as a ceRNA competitively bound to miR-21 to inhibit the function of miR-21 on promoting the biological progression of CRC. Furthermore, we found that miR-21 could bind to the mRNA of LIFR, a leukemia inhibitory factor receptor, and decrease the expression level of it. It was reported that the high expression of LIFR stimulated melanoma cell migration [36] and LIFR negatively regulated the PI-3K/AKT pathway in hepatocellular carcinoma and could function as a metastasis suppressor [18]. GAS5 could suppress the decrease of LIFR caused by miR-21 and rescue the function of LIFR on tumor cell viability. Many studies proved LIFR could repress some tumor, and our study was the first to prove miR-21 could suppress the mRNA of LIFR to promote the tumor progression.

The interactions of lncRNA, miRNA, and mRNA regulated the gene expression and protein function. Especially for tumor cells with abnormal cell physiology, revealing the mechanism of the interaction network was significant for the control and target treatment. Our study revealed a regulation network among GAS5, miR-21, and LIFR, and we found that GAS5 could bind to miR-21 to decrease the miR-21 level in tumor cells, so that the binding between miR-21 and LIFR was decreased, and as a result, the expression of LIFR increased and promoted the apoptosis of tumor cells. It was not the only pathway for GAS5, miR-21, and LIFR to inhibit the tumor cells, and one study reported that overexpression of GAS5 could inhibit cell proliferation and promote apoptosis by inhibiting miR-182-5p expression [24]. Our study first found that GAS5 was the lncRNA of miR-21 and it was meaningful to explain the function of miR-21. In addition, we found that LIFR was a target gene regulated by miR-21, and LIFR also could promote the apoptosis of tumor cells. It was reported that LIFR promoted tumor angiogenesis by upregulating IL-8 levels in colorectal cancer [16].

In conclusion, our study revealed a novel pathway that lncRNA GAS5 could suppress proliferation and metastasis of CRC by target miR-21/LIFR axis and provided a target for the study on treatment of CRC (Figure 7).

## Figures and Tables

**Figure 1:** Low expression of GAS5 in colorectal cancer (CRC) promotes the tumor metastasis and decreases the survival of patients. (a) Expression level of GAS5 in CRC tumor tissues lower than adjacent tissues. 53 Chinese CRC patient's specimens were detected by qPCR. (b) Low expression level of GAS5 decreases the survival of CRC patients. (c) Metastasis tissues had lower expression level of GAS5 than nonmetastasis tissues. (d) CRC cell lines including HCT-116, HT-29, SW480, LoVo, Caco-2, and LS174 t had lower expression of GAS5 than colorectal cell line NCM460 cells. ^*∗*^*P* < 0.05, ^*∗∗*^*P* < 0.01, ^*∗∗∗*^*P* < 0.001. Error bars indicate mean ± SD.

**Figure 2:** Knockdown of GAS5 increases colorectal cancer cells viability, inhibits apoptosis, and promotes migration. (a) Knockdown of GAS5 by specific siGAS5 and upregulation of GAS5 by transfection of plasmid carried GAS5 in SW480 cells. (b) Cell viability detected when SW480 cells were treated post 6 h, 24 h, 48 h, and 72 h by siGAS5, plv-GAS5, and NC. The absorbance value of each group was determined at a wavelength of 450 nm. (c) Cell apoptosis detected by flow cytometry through Annexin V-FITC/PI staining. Each group was assayed in a 96-well plate in triplicate. (d) Migration of cells was evaluated using transwell chambers at 24 h after transfection. ^*∗*^*P* < 0.05, ^*∗∗*^*P* < 0.01, ^*∗∗∗*^*P* < 0.001.

**Figure 3:** Knockdown of CAS5 promotes the tumor growth and the lesion of colorectal in the animal model. SW480 cells having different GAS5 expression status were injected into female BALB/C nude mice to analyze the effect on tumor. (a) Tumor weight detected in the BALB/C nude mice model after injection 15 days. (b) The colorectal of each group collected to analyze the tumor formation and metastasis by HE staining. (c) Statistics of lesion of colorectal. (d) Bodyweight. ^*∗*^*P* < 0.05, ^*∗∗*^*P* < 0.01, ^*∗∗∗*^*P* < 0.001.

**Figure 4:** GAS5 is suppressed by miR-21 in colorectal cancer cells to promote the CRC. (a) The potential binding sites between miR-143 and PVT1. (b) Expression levels of miR-21 decreased in all examined colorectal cancer cells. (c) The expression level of miR-21 increased in CRC cells transfected with siGAS5 as compared with those transfected with NC. (d) the cells cotransfected (e) and Western blot assays (f) with GAS5-WT and miR-21 mimic be detected. (g) Flow cytometry analyses of apoptosis rates of the transfected CRC cells at 72 h. (h) Colony formation assays conducted to measure the ability of cell survival in the transfected CRC cells. ^*∗*^*P* < 0.05, ^*∗∗*^*P* < 0.01, ^*∗∗∗*^*P* < 0.001.

**Figure 5:** GAS5 suppressed the inhibition of miR-21 on LIFR. (a) Bioinformatics prediction of miR-21 binding sites in LIFR 3′UTR sequence using miRBase. (b) Relative luciferase activities of wild-type (WT) and mutated (MUT) LIFR 3′UTR reporter plasmid in CRC cells cotransfected with miR-21 mimic. (e)-(f) LIFR protein levels coincided with the change of mRNA levels in NC and GAS5-miR-21 overexpressing cells. ^*∗*^*P* < 0.05, ^*∗∗*^*P* < 0.01, ^*∗∗∗*^*P* < 0.001.

**Figure 6:** GAS5 could rescue the inhibition of LIFR to suppress the tumor cells. (a) The effects of LIFR, siLIFR, GAS5+siLIFR, and miR-21+LIFR on cell activity levels in CRC cells. (b) Flow cytometry analyses of apoptosis rates of the transfected CRC cells at 72 h. (c) Colony formation assays conducted to measure the ability of cell survival in the transfected CRC cells. (d) The effects of LIFR, siLIFR, GAS5+siLIFR, and miR-21+LIFR on cleaved caspase-3 expression detected by WB. ^*∗*^*P* < 0.05, ^*∗∗*^*P* < 0.01, ^*∗∗∗*^*P* < 0.001.

**Figure 7:** Graphic summary of this study of lncRNA GAS5 suppressing proliferation and metastasis of CRC by target miR-21/LIFR axis.

**Table 1:** Characteristics of CRC patients.

Characteristics	Variable	Number (%)
Age (years)	Range (means ± SD)	35–62 (52 ± 6)

Gender	Male	26 (49.1)
	Female	27 (50.9)

Family history	No	40 (75.5)
	Yes	13 (24.5)

**Table 2:** The primers used in qRT-PCR.

Gene	Primer	Sequences
GAPDH	F	5′-GTCAACGGATTTGGTCTGTATT-3′
	R	5′-AGTCTTCTGGGTGGCAGTGAT-3′

U6	F	5′-CTCGCTTCGGCAGCACA-3′
	R	5′-AACGCTTCACGAATTTGCGT-3′

GAS5	F	5′-CAGACGTGTGCTCTTC-3′
	R	5′-CGATCTGTAAGTCCACCA-3′

miR-21	F	5′-TGCCTCCCCGACACCATG-3′
	R	5′-GGATTCCCAGCCATTGTCC-3′

LIFR	F	5′-TGGAACGACAGGGGTTCAGT-3′
	R	5′-GAGTTGTGTTGTGGGTCACTAA-3′

## Data Availability

The datasets used and/or analyzed during the present study are available from the corresponding author upon request.
